# Relationship between Prognosis with Dynamic Changes of Thyroid Hormone and Cortisol Hormone in Patients with Severe Craniocerebral Injury

**DOI:** 10.1155/2022/1883107

**Published:** 2022-09-19

**Authors:** Chuang Ding, Jianbo Liu, Kejun Liu, Xiaoteng Yao

**Affiliations:** Department of Neurosurgery, Huizhou First People's Hospital, Huizhou, China

## Abstract

**Objective:**

To analyze the dynamic changes of thyroid hormone and cortisol hormone (COR) and their relationship with prognosis in patients with severe craniocerebral injury.

**Methods:**

A retrospective analysis of 48 patients with severe craniocerebral injury who were admitted to our hospital from January 2014 to January 2017 was performed. According to the Glasgow Outcome Scale (GOS) after 3 months of treatment, the patients were divided into a favorable prognosis group (GOS score = 4-5) and a poor prognosis group (GOS score = 1–3). Clinical data such as ICU hospitalization time and mechanical ventilation time between the two groups were collected and compared. The GCS score was evaluated and recorded at 24 h and 7 d after injury, respectively. The fasting venous blood was collected from patients at 24 h and 7 d after injury, and the levels of thyrotropin (TSH), total triiodothyronine (TT3), total thyroxine (TT4), free triiodothyronine (FT3), and free thyroxine (FT4) were detected by the time-resolved fluorescence immunoassay, while the cortisol (COR) levels were examined by the chemiluminescence assays. The prognostic risk factors of patients with severe craniocerebral injury were analyzed using logistic regression analysis. A nomogram prediction model was constructed based on the results of the logistic analysis. The value of each factor in predicting the prognosis of patients with severe craniocerebral injury was analyzed using the ROC curve.

**Results:**

Significant differences existed between the poor prognosis group and the favorable prognosis group in age, whether complicated with a cerebral hernia, intracranial hematoma volume, admission time, ICU hospitalization time, GCS score, and mechanical ventilation time (*P* < 0.05). At 24 h after injury, the levels of TT4, FT3, and FT4 in the poor prognosis group were significantly lower than those in the favorable prognosis group (*P* < 0.05). On the 7^th^ day after the injury, the levels of FT3, FT4, TT3, TT4, and TSH in the poor prognosis group were prominently lower than those in the favorable prognosis group (*P* < 0.05). At 24 h after injury, the COR level in the poor prognosis group was observably higher than that in the favorable prognosis group (*P* < 0.05). Logistic regression analysis showed that age, complicated with a cerebral hernia, length of stay in ICU, FT3, FT4, TT4, and COR were the risk factors affecting the prognosis of patients with severe craniocerebral injury (*P* < 0.05), while the GCS score was the protective factor (*P* < 0.05). ROC curve analysis revealed that the area under the curve (AUC) of ICU length of stay, GCS score, FT3, and FT4 to predict the prognosis of patients with severe craniocerebral injury was better with 0.841, 0.885, 0.881, and 0.850, respectively. The survival curve drawn by the K-M method showed that high levels of serum FT3, FT4, and TT4 and low levels of COR were conducive to improve the overall survival time of patients (*P* < 0.05).

**Conclusion:**

Abnormal levels of thyroid hormone and cortisol hormone were found in patients with severe craniocerebral injury. Age, combined brain herniation, ICU length of stay, FT3, FT4, TT4, COR, and GCS scores were all prognostic factors in patients with severe traumatic brain injury. These factors have high value in judging the death and survival of patients with severe craniocerebral injury.

## 1. Introduction

Severe craniocerebral injury is a traumatic disease with a high clinical incidence rate. With the rapid development of industry and transportation in recent years, the incidence rate of severe craniocerebral injury is increasing year by year, seriously endangering the life and health of patients [1]. Previous statistics show that the mortality and disability rates of patients with severe craniocerebral injury are as high as 27% and 53%, respectively, which not only loads great pain to patients but also aggravates the economic burden on families and the social economy [2, 3]. Recent studies have found that patients with craniocerebral injury have serious neuroendocrine disorders, including water and sodium balance disorders, microenvironment changes, abnormal circulatory function, and energy metabolism, which induce abnormal hypothalamic-pituitary-thyroid axis function and aberrant thyroid-related hormone secretion. Thyroid hormone can mediate almost all human cells, participate in the body growth and development, body metabolism, and organ activities, and maintain the excitability of the nervous system. The aberrant level of thyroid-related hormones further damages the function of neurogenic multiple organs such as the heart, lung, and kidney, which eventually aggravates the neuroendocrine disorder of patients, and even leads to death [4, 5]. In addition, severe craniocerebral injury can also abnormally activate the hypothalamic-pituitary-adrenal axis of the body and stimulate the production of cortisol (COR). COR is an adrenocortical hormone secreted from the adrenal cortex, which mediates the metabolic process of sugars. COR can also affect the changes and metabolism of systemic hormones and the functional changes of systemic organs [6]. The present study retrospectively analyzed the clinical data of 48 patients with severe craniocerebral injury treated in our hospital from January 2014 to January 2017, and the dynamic changes of thyroid hormone and COR, as well as their relationship with prognosis in patients with severe craniocerebral injury.

## 2. Materials and Methods

### 2.1. General Materials

A total of 48 patients with severe craniocerebral injury treated in our hospital from January 2014 to January 2017 were selected as the subjects. Inclusion criteria were as follows: (1) all patients were treated in the Intensive Care Department of our hospital. The initial Glasgow Coma Scale (GCS) was ≤ 13. The patients had intracranial hemorrhagic lesions, acute hypopituitarism, and traumatic brain injury, which were confirmed by CT and MRI; (2) patients aged between 18 and 65 years old; (3) patients with more than one week survival time; (4) patients and the family members had the good compliance to the examination and treatment and signed the informed consent form. Exclusion criteria were as follows: (1) patients with consciousness disorder caused by previous nervous system or patients with mental diseases, severe disability, or patients in a vegetative state; (2) patients with diabetes, hypothyroidism or hypocortisolism, intracranial hypertension, optic papilledema, and other diseases history; (3) pregnant patients; (4) patients complicated with the malignant tumor within five years; (5) patients with serious dysfunction of important organs history. According to the GOS after 3 months of treatment, the patients were divided into a favorable prognosis group (GOS score = 4-5) and a poor prognosis group (GOS score = 1–3). There were 13 cases in the poor prognosis group, including 6 males and 7 females, with an average age of (45.67 ± 25.10) years. There were 35 cases in the favorable prognosis group, including 20 males and 15 females, with an average age of (48.50 ± 19.29) years. There was no significant difference in age and sex between the two groups (*P* < 0.05). The general material selection process was shown in Figure 1.

### 2.2. Outcome Measures

#### 2.2.1. Clinical Indicators

The responsible nurses asked the patients or their families to collect general information such as age, gender, and admission time of the two groups of patients, and closely observed the patients' conditions. The nurses also observed and recorded whether the two groups of patients were complicated with brain herniation, intracranial hematoma volume, cerebral contusion range, intracranial hematoma location, ICU stay time, and mechanical ventilation time. The patient's GCS scores were evaluated and recorded at 24 h and 7 d after injury, respectively. The GCS score is a clinical scale for assessing the disturbance of consciousness in patients, which includes three components, eye-opening response, verbal response, and motor response. Scores range from 0 to 15, with lower scores indicating a more severe disturbance of consciousness.

#### 2.2.2. Serum Indicators

The levels of thyroid-stimulating hormone (TSH), total triiodothyronine (TT3), total triiodothyronine (TT4), free triiodothyronine (FT3), and free thyroxine (FT4) were detected by time-resolved fluoroimmunoassay. The changes in COR levels in each group were detected by chemiluminescence.

#### 2.2.3. Resolved Fluorescence Immunoassay

The fasting venous blood in the morning of 24 h and 7 d after injury was collected from the two groups and centrifuged at 3000 r/min for 30 min. The serum was carefully separated and frozen at −80°C for standby. The sample was mixed with tris-HCL solution containing Eu^3+^ with a pH of 7.8 in the ratio of BCPDA : Eu^3+^ = 1 : 1 and the mixture took a warm bath at 37°C for 1 h. 5 ml solution and the blank solution as the reference was prepared. The sample was added to the 1 cm cuvette and was measured with the absorbance of 325 nm on the UV-V spectrophotometer.

#### 2.2.4. Chemiluminescence Method

The fasting venous blood in the morning of 24 h and 7 d after injury was collected from the two groups and centrifuged at 3000 r/min for 30 min. The serum was carefully separated and frozen at −80°C for standby. The tested serum was put into the automatic chemiluminescence immunoassay analyzer TESMI i200 (Shanghai Toujing Life Technology Co., Ltd., Shanghai, China) for chemiluminescence detection. Open the BPCL measurement program, click the “regulation” item in the menu list to display the drop-down menu, click the set parameter command to input the temperature and high-pressure values, click the display environment window command box to display the temperature and high-pressure values, and use the command in the control menu to set the temperature and high-pressure values to meet the conditions suitable for the experiment.

#### 2.2.5. Follow-Up

All patients were followed up for 4 years, the start time of follow-up was the time of admission in our hospital, and the end time was January 2021. Follow-up was conducted through an outpatient clinic or by telephone. The overall survival time of patients was recorded and compared.

### 2.3. Statistical Analysis

Spss20.0 software was used to analyze the experimental data. The measurement data such as age, GCS score, TT3, admission time, and ICU length of stay were in line with normal distribution and homogeneity of variance, expressed as ($\bar{x}$ ± *s*), and compared using a *t*-test. The enumeration data such as gender were expressed in (%), and compared using *χ*^2^ inspection. The correlation between serum-related indexes and GCS score was analyzed by Pearson correlation. The prognostic risk factors in patients with severe craniocerebral injury were determined by the logistic regression analysis and a nomogram model was constructed. The value of various factors in predicting the prognosis of patients with severe craniocerebral injury was conducted by the ROC curve analysis. The Kaplan–Meier survival curve was used to analyze the relationship between the levels of thyroid hormone and cortisol and the survival rate of patients with severe traumatic brain injury. *P* < 0.05 was taken as statistically significant.

## 3. Results

### 3.1. Relationship between Clinical Characteristics and Prognosis in 48 Patients with Severe Craniocerebral Injury

Compared with the favorable prognosis group, the patients in the poor prognosis group had significantly higher levels of age ≥ 60 years old, combined with brain herniation, intracranial hematoma volume ≥ 50 ml, admission time, ICU stay time, GCS score, and mechanical ventilation time (*P* < 0.05, Table 1).

### 3.2. Relationship between Dynamic Changes of Thyroid Hormones with Prognosis

At 24 h after injury, the levels of TT4, FT3, and FT4 in the poor prognosis group were significantly lower than those in the favorable prognosis group. At 7 d after injury, the levels of FT3, FT4, TT3, TT4, and TSH in the poor prognosis group were significantly lower than those in the favorable prognosis group (*P* < 0.05, Table 2).

### 3.3. Relationship between Dynamic Changes of COR with Prognosis

At 24 hours after injury, the level of COR in the poor prognosis group was significantly higher than that in the favorable prognosis group (*P* < 0.05), while there was no significant difference in the COR level between the two groups at 7 d after injury (*P* < 0.05, Table 3).

### 3.4. Logistic Regression Analysis of Prognostic Risk Factors in Patients with Severe Craniocerebral Injury

The poor/favorable prognosis of patients was taken as the dependent variable, and the statistically significant factors were included in the logistic regression model as the independent variables for regression analysis. Logistic regression analysis showed that age, concomitant brain herniation, ICU length of stay, FT3, FT4, TT4, and COR were the risk factors affecting the prognosis of patients with severe craniocerebral injury (*P* < 0.05), and GCS score was the protective factor (*P* < 0.05, Table 4).

### 3.5. Establishment of Nomograph Model for Predicting Prognosis Risk of Severe Craniocerebral Injury

Based on the results of multivariate Logistic regression analysis, the age, concomitant brain herniation, ICU length of stay, FT3, FT4, TT4, COR, and GCS were included as the factors to build a prognosis risk prediction model for severe craniocerebral injury. Each influencing factor was compared with the score scale to obtain a separate score, and the sum of the scores was compared with the total score scale of the nomogram. The higher the total score was, the higher the risk of poor prognosis was. The model consistency coefficient was 0.826, with high internal consistency. The validation results of the ROC curve showed that the area under the curve of the model for predicting the prognosis of severe traumatic brain injury was 0.834 (95% CI: 0.736–0.933), the sensitivity was 87.50%, and the specificity was 80.00% (Figures 2–4).

### 3.6. Value of ROC Curve Analysis in Predicting Prognosis of Patients with Severe Craniocerebral Injury

The results of the ROC curve analysis showed that the area under the curve (AUC) of ICU length of stay, GCS score, FT3, and FT4 was well for predicting the prognosis of patients with severe traumatic brain injury, with 0.844, 0.807, 0.838, and 0.867, respectively (Table 5 and Figure 5).

### 3.7. Relationship between Thyroid Hormone and Cortisol Levels and Survival Time of Patients with Severe Craniocerebral Injury

The survival rate of 48 patients from operation to death or the last follow-up date was recorded, and the survival rate was 58.33% (28/48). The results of the survival curve drawn by the K-M method showed that high levels of serum FT3, FT4, TT4, and low levels of COR were beneficial to improve the overall survival of patients (Table 6 and Figure 6).

## 4. Discussion

Severe craniocerebral injury is one of the trauma diseases with a high incidence rate in the world, which poses a serious threat to human health due to its highest mortality and disability rate of all trauma [7, 8]. Cerebral ischemia and hypoxia are common pathophysiological changes in secondary injury after brain injury, and the degree of ischemia is closely related to the prognosis. Therefore, the key to improve the prognosis of patients with brain injury is to control the secondary ischemic injury after primary brain injury.

Although great progress in the diagnosis and treatment of severe craniocerebral injury has been made due to the rapid development of medical technology, the incidence of poor prognosis is still high [9]. Here, the incidence of poor prognosis in 48 patients with severe craniocerebral injury was 27.08%, indicating the mortality and fatality rate of patients with severe craniocerebral injury were still high, although various comprehensive treatment measures including surgery have been taken. Therefore, how to improve the rescue success rate and prognosis of patients with severe craniocerebral injury has become a subject to be further studied and solved.

Previous studies have found that the function of the hypothalamic-pituitary-thyroid axis changes after severe craniocerebral injury, mainly manifested as hypothyroidism. Under normal circumstances, there is a certain dynamic balance between FT3 and FT4, and TT3 and TT4 in the blood circulation. FT3 and FT4 play their biological role by entering the target cells [10]. When the brain is seriously injured, intracranial hemorrhage induces an increase in intracranial pressure, ischemia, and hypoxia in brain tissue. At the same time, the activities of 5-deiodinase and nerve cell enzymes are greatly reduced, resulting in a decrease in the number of TT3 and the intake of TT4 [11, 12]. At the same time, a severe craniocerebral injury may also induce the occurrence of stress diseases, thus, inhibiting the secretion of TSH and reducing the level of TSH [13]. Recent studies have found that patients with craniocerebral injury are accompanied with cerebral infarction, cerebral thrombosis, and other complications, which indirectly or directly damage the hypothalamus, pituitary, and other parts of the body to affect the secretion of hormones such as COR. Obviously aberrant COR level may induce an increase in intracranial pressure, cerebral infarction, hypoxemia, and other conditions, aggravating the patient's condition [14]. In this experiment, the levels of FT3, FT4, TT3, TT4, TSH, and COR in the poor prognosis group were significantly lower than those in the favorable prognosis group at 24 h and 7 d after injury, which suggested that abnormally expressed thyroid hormone and cortisol hormone might be related to the prognosis of patients with severe craniocerebral injury. Relevant data show that the degree of injury in patients with traumatic brain injury can be assessed by estimating the levels of thyroid-related hormones and cortisol in the clinical diagnosis and treatment of severe traumatic brain injury, and it is highly scientific for evaluating treatment effects, treatment risks and related issues [15, 16]. Therefore, this study speculated that the thyroid-related hormone level and cortisol changes could be used as sensitive indicators to evaluate the prognosis of severe craniocerebral injury, and the following study would be carried out.

Severe craniocerebral injury has rapid progress and poor prognosis, which seriously threatens people's life and health. Early assessment of the prognosis of severe craniocerebral injury and targeted intervention are of great significance in improving the prognosis and reducing the mortality of patients [17]. GCS score is a commonly used clinical scale to evaluate the changes of consciousness of ICU patients with good validity and has a certain value in evaluating the neurological function and prognosis of patients with severe craniocerebral injury [18]. In order to further analyze the relationship between the changes in thyroid hormone and COR levels and the prognosis of patients with severe craniocerebral injury, a logistic regression model was used for regression analysis. The results showed that age, concomitant brain herniation, ICU length of stay, FT3, FT4, TT4, and COR were the risk factors (*P* < 0.05), and GCS score was the protective factor affecting the prognosis of patients with severe craniocerebral injury (*P* < 0.05). The AUC of ICU length of stay, GCS score, FT3, and FT4 for predicting the prognosis of patients with severe traumatic brain injury was better (all >0.8), indicating that the level of thyroid hormone and cortisol hormone changed significantly in patients with severe traumatic brain injury with poor prognosis. Monitoring dynamic changes are helpful to assess the prognosis of patients. Some scholars have found that the more severe the condition of patients with severe craniocerebral injury is, the greater the change range of thyroid hormone level and cortisol is [19]. The contents of TT3, FT3, and COR can be used as indicators to evaluate the prognosis of patients with craniocerebral injury. It can be seen that the changes of thyroid-related hormones and cortisol can not only reflect the degree of brain tissue damage in patients with severe brain injury but also play a guiding role in the clinical treatment and prognosis evaluation of brain injury. In addition, based on the multivariate Logistic regression analysis results, the risk prediction model for the prognosis of severe traumatic brain injury constructed in this study had a good degree of discrimination, suggesting that the nomogram in this study could be used as a good tool for evaluating the prognosis of severe traumatic brain injury. The results of the K-M survival curve showed that high levels of serum FT3, FT4, TT4, and low levels of COR were beneficial to improve the overall survival of patients. It has been shown that severe craniocerebral injury causes significant changes in thyroid secretion function [20]. Evaluation of treatment outcomes, treatment risks, and related issues by predicting changes in thyroid hormones and cortisol, is highly scientific. In the present study, high levels of serum FT3, FT4, TT4, and low levels of COR were independent risk factors affecting the prognosis of patients with severe craniocerebral injury, which suggested that these indicators could act as markers for the detection of severe brain injury in the early diagnosis and treatment of patients.

In conclusion, the levels of thyroid hormone and cortisol hormone in patients with severe craniocerebral injury are significantly abnormal. Age, combined brain herniation, ICU length of stay, FT3, FT4, TT4, COR, and GCS scores are all prognostic factors in patients with severe craniocerebral injury. High levels of serum FT3, FT4, TT4, and low levels of COR are beneficial to improve the overall survival of patients. These factors have high value in judging the death and survival of patients with severe craniocerebral injury. However, due to the short research time and the small number of samples in this experiment, the experimental results may have certain deviations. In the future, the experimental objects and research time will be expanded for in-depth research.

## Figures and Tables

**Figure 1:** Process of general materials selection.

**Figure 2:** Nomograph analysis.

**Figure 3:** Calibration curve.

**Figure 4:** ROC curve.

**Figure 5:** The value of ROC curve analysis of various factors in predicting the prognosis of patients with severe craniocerebral injury.

**Figure 6:** K-M survival curve of patients with severe craniocerebral injury. (a) Survival curves at different FT3 levels; (b) survival curves at different FT4 levels; (c) survival curves at different TT4 levels; (d) survival curves at different COR levels.

**Table 1:** Relationship between clinical characteristics and prognosis in 48 patients with severe craniocerebral injury (%, *x* ± *s*).

Factors		The favorable prognosis group (*n* = 35)	The poor prognosis group (*n* = 13)	*t*/*χ*^2^	*P* value
Gender	Male	20 (57.14)	6 (46.15)	0.461	0.497
	Female	15 (42.86)	7 (53.85)		

Age (year)	<60	33 (94.29)	9 (69.23)	5.441	0.020
	≥60	2 (5.71)	4 (30.77)^*∗*^		

Cerebral hernia	Yes	10 (28.57)	8 (61.54)^*∗*^	4.396	0.036
	No	25 (71.43)	5 (38.46)		

Intracranial hematoma volume	<50 ml	24 (68.57)	4 (30.77)	5.573	0.018
	≥50 ml	11 (31.43)	9 (69.23)^*∗*^		

Admission time (h)		3.8 ± 1.1	6.5 ± 2.1^*∗*^	5.813	<0.001

Cerebral contusion and laceration range	Single	20 (57.14)	5 (38.46)	1.326	0.250
	Multiple	15 (42.86)	8 (61.54)		

Location of intracranial hematoma	Epidural hematoma	17 (48.57)	5 (38.46)		
	Intradural hematoma	11 (31.43)	4 (30.77)	1.284	0.733
	Intracerebral hematoma	5 (14.29)	2 (15.38)		
	Mixed hematoma	2 (5.71)	2 (15.38)		

ICU hospitalization time (d)		9.0 ± 2.6	16.9 ± 5.3^*∗*^	6.402	<0.001

GCS score (score)	24 h after injury	10.00 ± 0.12	9.75 ± 0.29^*∗*^	4.264	<0.001
	7 days after injury	13.16 ± 1.97	9.71 ± 3.45^*∗*^	4.346	<0.001

Mechanical ventilation time (d)		1.05 ± 0.26	3.01 ± 0.46^*∗*^	18.608	<0.001

*Note.* ^*∗*^ is compared with the favorable prognosis group, ^*∗*^*P* < 0.05.

**Table 2:** Relationship between dynamic changes of thyroid hormones with prognosis ($\bar{x}$ ± *s*).

Index	Time	The favorable prognosis group (*n* = 35)	The poor prognosis group (*n* = 13)	*t*	*P value*
FT3	24 h after injury	3.80 ± 0.35	3.39 ± 075^*∗*^	2.591	0.012
(pmol/L)	7 d after injury	3.92 ± 0.58	3.53 ± 0.30^*∗*^	2.301	0.025
FT4	24 h after injury	17.73 ± 4.49	11.52 ± 9.23^*∗*^	3.137	0.003
(pmol/L)	7 d after injury	15.56 ± 2.96	14.63 ± 2.62^*∗*^	3.239	0.002
TT3	24 h after injury	1.21 ± 0.55	1.19 ± 0.61^*∗*^	0.108	0.913
(pmol/L)	7 d after injury	1.48 ± 0.13	1.12 ± 0.27^*∗*^	6.244	<0.001
TT4	24 h after injury	130.03 ± 43.30	98.28 ± 29.04^*∗*^	2.439	0.018
(pmol/L)	7 d after injury	110.90 ± 4.85	103.13 ± 5.78^*∗*^	4.682	<0.001
TSH	24 h after injury	0.93 ± 0.84	0.83 ± 0.86	0.364	0.717
(pmol/L)	7 d after injury	1.29 ± 0.23	0.71 ± 0.97^*∗*^	3.347	0.002

*Note.* ^*∗*^ is compared with the favorable prognosis group, ^*∗*^*P* < 0.05.

**Table 3:** Relationship between dynamic changes of COR with prognosis ($\bar{x}$ ± *s*).

Groups	COR (pmol/L)	
	24 h after injury	7 d after injury
The favorable prognosis group (*n* = 35)	424.43 ± 152.38	410.12 ± 128.15
The poor prognosis group (*n* = 13)	541.29 ± 159.41 ^*∗*^	412.90 ± 158.88
*T*	2.332	0.062
*P*	0.024	0.950

*Note.* ^*∗*^ is compared with the favorable prognosis group, ^*∗*^*P* < 0.05.

**Table 4:** Logistic regression analysis of prognostic risk factors in patients with severe craniocerebral injury.

Factors	*B*	SE	Wald	*P*	OR	95%CI
Age	0.988	0.351	8.033	**0.001**	2.676	1.313∼5.421
Cerebral hernia	1.872	0.369	13.465	0.001	6.552	3.015∼14.280
Intracranial hematoma volume	0.652	0.362	4.977	0.085	1.910	0.935∼3.829
Admission time (h)	0.007	0.008	3.506	0.105	1.008	0.995∼1.019
ICU hospitalization time (d)	0.670	0.359	5.194	**0.022**	1.890	0.982∼4.036
GCS score (score)	–1.189	0.352	9.713	**0.001**	0.315	0.150∼0.629
Mechanical ventilation time (d)	0.528	0.389	2.714	0.113	1.256	0.772∼1.398
FT3	1.378	0.371	9.986	**0.001**	4.025	1.927∼8.172
FT4	1.023	0.359	7.930	**0.001**	2.815	1.372∼5.6060
TT3	0.939	0.352	2.725	0.089	1.262	0.857∼1.369
TT4	1.263	0.370	9.226	**0.001**	3.852	1.856∼8.816
TSH	0.688	0.575	2.079	0.115	1.025	1.001∼1.358
COR	1.285	0.369	9.449	**0.001**	3.642	1.625∼7.346

**Table 5:** Value of ROC curve analysis in predicting prognosis of patients with severe craniocerebral injury.

Factors	AUC	Sensitivity	Specificity	*P value*	95% CI
Age	0.759	75.00	64.00	<0.001	0.633∼0.846
Cerebral hernia	0.781	77.50	70.00	<0.001	0.682∼0.886
ICU hospitalization time (d)	0.844	82.50	73.40	<0.001	0.748∼0.935
GCS score	0.807	88.50	78.60	<0.001	0.815∼0.955
FT3	0.838	88.00	79.20	<0.001	0.804∼0.958
FT4	0.867	90.50	76.40	<0.001	0.754∼0.946
TT4	0.722	80.40	74.60	<0.001	0.616∼0.840
COR	0.701	74.30	69.50	0.002	0.600∼0.833

**Table 6:** difference in survival time of thyroid hormone and cortisol levels.

Factors	*P*	HR	95%CI
FT3 ≥ 3.8 vs FT3 < 3.8	<0.001	29.030	25.015∼33.044
FT4 ≥ 13.6 vs FT4 < 13.6	<0.001	32.853	29.721∼35.986
TT4 ≥ 110.5 vs TT4 < 110.5	<0.001	34.546	32.366∼36.725
COR < 325.1 vs COR ≥ 325.1	<0.001	33.696	30.200∼37.191

## Data Availability

All data, models, and code generated or used during the study appear in the submitted article.
